The article "Can combined compost and biochar application improve the quality of a highly weathered coastal savanna soil?" was published in 2021. Journal: Heliyon.

# Can combined compost and biochar application improve the quality of a highly weathered coastal savanna soil?

**DOI:** 10.1016/j.heliyon.2021.e07089

**Published:** 2021-05-21

**Authors:** Kwame Agyei Frimpong, Emmanuel Abban-Baidoo, Bernd Marschner

**Affiliations:** a Department of Soil Science, School of Agriculture, College of Agriculture and Natural Sciences, University of Cape Coast, Cape Coast, Ghana; b Department of Soil Science and Soil Ecology, Institute of Geography, Ruhr University, Bochum, Germany

**Keywords:** Biochar, Co-compost, Soil quality, Microbial biomass, Basal respiration

## Abstract

Soil fertility decline is a major constraint to crop production in sub-Saharan Africa. The positive effect of biochar and compost applications on soil fertility has been reported by many authors. In this study, a 30-day laboratory incubation experiment was done using 120 g samples each of a Haplic acrisol amended with corn cob biochar (cbio), rice husk biochar (rbio), coconut husk biochar (coco300 and coco700) or poultry manure compost (compost); and co- composted rice husk biochar (rcocomp) or co-composted corn cob biochar (cococomp) at rates of 1 % w/w amendment: soil, respectively. Other treatments in the study were combined poultry manure compost and corn cob biochar or rice husk biochar (1 % compost + 1% biochar: 1% soil w/w), respectively, to examine their effects on basal soil respiration, soil pH; soil microbial carbon; cation exchange capacity; total organic carbon, total nitrogen and available nitrogen concentration. Biochar and compost applied solely or together, and composted biochar increased soil pH by 0.28–2.29 pH units compared to the un-amended control. Basal respiration from the sole compost or composted rice husk, or corn cob biochar or combined biochar and compost were higher than the un-amended control, which was similar to that from the biochar only treatments. TOC in the sole compost and combined corn cob biochar and compost treatments were up to 37% and 117% higher, respectively, than the control. Combined application of rice husk biochar and compost increased MBC by 132% while sole compost addition increased MBC by 247%, respectively, compared to the control. In conclusion, the study demonstrated that sole or combined application of compost and biochar, or composted biochar improved soil quality parameters such as soil pH and MBC, and promoted soil C stabilization through enhanced TOC and reduced soil C loss through basal respiration.

## 1 Introduction

Improving soil quality is critical to increasing crop yields, combating rural poverty and reversing natural resource degradation in sub-Saharan Africa (SSA) (Vanlauwe et al., 2015). Biochar, a highly stable, aromatic carbon by-product obtained from the pyrolysis of organic materials at relatively low temperatures (<700 °C) in the presence of low or no oxygen, has been shown to be an effective amendment to improve soil quality (Lehmann et al., 2011). Biochar is not biologically inert but follows a biphasic mineralization pattern where the more labile compounds are rapidly mineralized first, after which the recalcitrant carbon degrades more slowly (Cross and Sohi, 2011). Consumption of labile compounds from biochar decomposition changes soil physicochemical characteristics (Lehmann et al., 2011) and soil biological parameters including basal soil respiration and microbial biomass (Bailey et al., 2011; Durenkamp et al., 2010). Although, the rate of biochar decomposition is slower than other soil carbon pools, it can provide similar soil ecological services including nutrient and water retention as other organic materials (Atkinson et al., 2010). Kolb et al. (2009) reported that the specific surface area of biochar, which is approximately 200–400 m^2^ g^−1^, is comparable to that of the soil clay fraction. Thus, biochar addition can increase the specific surface area of soil (Arthur et al., 2015), increase water and air availability and stimulate microbial activity for enhanced soil quality.

The article "Can combined compost and biochar application improve the quality of a highly weathered coastal savanna soil?" was published in 2021. Journal: Heliyon.

Soil acidity is a major constraint to crop production in many areas of tropical Africa. Liming is the conventional option for soil acidity mitigation, but lime is costly and scarcely available to smallholder farmers in SSA hence its adoption is very low. Van Zweiten et al. (2010) found that biochar added to soil exerts a liming effect, which can promote nutrient release from native soil nutrients pools. According to Oguntunde et al. (2004), the basic metallic ions contents of the ash component of the biochar applied can decrease soil acidity and create a growth-stimulating effect, especially in soils with low fertility (Jones et al., 2012). Biochar application has potential to promote soil C and N retention, increase cation exchange capacity and reduce anthropogenic greenhouse gas (CO_2_, N_2_O and CH_4_) emissions (Sohi et al., 2010; Singh et al., 2010).

Compost produced from aerobic decomposition of organic materials has been shown to have significant effects on soil physicochemical properties (Tibu et al., 2019). For instance, composts produced from crop residues, manures and other biomass waste products can increase soil nutrient content (Agromisa et al., 2005). Thus, application of composts is a commonly recommended practice that can introduce nutrients to soil and improve yields in low-input farming systems in SSA. However, under the high temperature and rainfall conditions prevailing in SSA, composts are rapidly mineralized within months or a few years after soil application (Schulz et al., 2013) and the nutrients released may be subjected to leaching or gaseous losses.

The article "Can combined compost and biochar application improve the quality of a highly weathered coastal savanna soil?" was published in 2021. Journal: Heliyon.

Many biochars are N-poor but rich in stable C (Singh et al., 2010) while most compost are rich in nutrients including N. Combined biochar and compost application can compensate for the shortcomings of each other such that their interactive effect is likely to improve soil quality. Liu et al. (2012) observed a synergistic positive effect of compost and biochar mixtures on soil organic matter content, nutrients concentrations, and water-storage capacity of a sandy soil under field conditions. Similarly, Agegnehu et al. (2015) found that, application of compost and biochar improved soil water and nutrient retention as well as water and nutrients uptake by the plants. In their study, however, little or no synergistic effect was observed. Abudjabha et al. (2016) reported that application of biochar and compost enhanced microbial abundance due to enhanced formation of macropores and bioturbation. Biochar co-composting has been reported to minimize C (Czekała et al., 2016) and N losses (Kammann et al., 2015; Steiner et al., 2010), to decrease N_2_O (Wang et al., 2013) and CH_4_ (Chowdhury et al., 2014) emissions compared to composting without biochar but the high diversity of biochar feedstocks makes it quite difficult to draw general conclusions on biochar co-composting effects.

The objective of the study was to examine the effect of compost and biochar, applied singly, in combination or co-composted on basal soil respiration, and soil quality indicators such as soil pH, soil microbial biomass carbon (MBC), Cation Exchange Capacity (CEC), Total Organic Carbon (TOC), Total Nitrogen (TN) and available N concentration. In previous studies biochars have often been applied singly or in combination with compost in their fresh forms. The novelty of this study is the inclusion of poultry manure co-composted with biochar produced from different feedstock to allow for an assessment of their effect on soil quality indicators compared with fresh additions of biochar and/or compost. The study was underpinned by the hypothesis that carbon-rich biochar and nitrogen-rich compost, applied together, can complement each other to improve soil quality indicators such as soil pH, C and N contents, soil microbial biomass and enhance soil C stabilization by minimizing soil C loss via respiration.

## 2 Materials and methods

### 2.1 Soil, compost, biochar and composted biochar

Surface (0–20 cm) soil collected from an arable field at the University of Cape Coast Teaching and Research farm in Ghana (5°07′N, 1°17′W) was used for the study. The soil sampling site is located in the humid, coastal savannah agro-ecological zone with a mean annual precipitation of 1400 mm and a mean temperature of 20 °C. The soils, which are developed on sandstones, shales and conglomerates are classified as a Haplic acrisol (IUSS Working Group WRB, 2015). The soil samples were collected from 20 different spots across a one hectare land, previously cropped with maize without any fertilization and bulked to form a composite sample for the study. The soil was well-drained and had a sandy loam texture (18, 9 and 73% clay, silt, and sand, respectively); with a pH of 4.39, electrical conductivity of 200 μS cm^−1^; total organic carbon of 9.3 g kg^−1^, total nitrogen of 0.73 g kg^−1^ and total phosphorus, potassium and magnesium contents of <0.4, 11.9, and 9.3 mg 100 g^−1^, respectively.

The article "Can combined compost and biochar application improve the quality of a highly weathered coastal savanna soil?" was published in 2021. Journal: Heliyon.

The corn cob and rice husk biochars were produced by slow pyrolysis at approximately 450 °C in a locally produced kiln under low oxygen conditions. The coconut husk biochar was pyrolysed in a muffle furnace at 300 and 700 °C, respectively. The composted biochars were produced during the *UrbanFood plus* project in Tamale, Northern Ghana. The basic components of the composted biochars included poultry manure (15 vol-%) and rice straw (60 vol-%) and either corn cob or rice husk biochar (25 vol-%) (Volker Haring, personal communication). The chemical properties of the soil and amendments used in the study are presented in Table 1.

**Table 1:** Chemical properties of amendments used in the study.

Amendment	pH	TN (%)	Moisture (%)	FC (%)	Ash (%)	VOM (%)
Rice husk biochar	7.2	0.75	9.85	44.26	20.1	25.79
Corn cob biochar	8.2	0.87	5.03	59.82	19.6	15.55
Coconut husk biochar (300 °C)	8.1	0.91	5.21	55.2	22.8	16.79
Coconut husk biochar (700 °C)	8.4	0.87	5.01	59.8	27.3	7.89
Composted rice husk biochar	8.5	0.92	5.04	43.7	29.6	21.66
Composted corn cob biochar	8.2	0.96	5.82	47.5	28.3	18.38
Rice husk compost	8	1.1	13.89	31.9	20.1	34.11

FC = fixed carbon, TN = total nitrogen, VOM = Volatile organic matter.

### 2.2 Experimental setup

A 30-day incubation experiment was conducted with a Haplic acrisol soil (0–20 cm) in Kilner jars (500 ml). Each jar was filled with 120 g air dry soils that had been sieved by mesh size of 2 mm. The soils were pre-incubated at 60% WHC and 25 °C for 10 days prior to addition of the amendments to re-initiate microbial activity after storage, and to minimise fluctuations in soil water content at the start of the experiment. At the end of the pre-incubation, the soils in each Kilner jar were mixed thoroughly with the appropriate type and quantity of soil amendment and adjusted to 60% WHC. Each treatment was replicated 3 times for basal respiration measurements on days 7, 14, 21 and 30, respectively. The soils were destructively sampled on day 30 for MBC, pH, TOC, TON and CEC analyses. The different treatments and the respective quantities of amendments mixed with the soil during incubation, as well as water soluble organic carbon content (WSOC) in each mixture are summarized in Table 2.

The article "Can combined compost and biochar application improve the quality of a highly weathered coastal savanna soil?" was published in 2021. Journal: Heliyon.

**Table 2:** Treatment details (amendments-soil mixtures).

Amendment	Quantity (g 120 g^−1^ soil)	WSOC (g kg^−1^)
Rice husk biochar (rbio)	1.2	0.54
Corn cob biochar (cbio)	1.2	0.43
Coconut husk biochar (300 °C) (coco300)	1.2	3.20
Coconut husk biochar (700 °C) (coco700)	1.2	3.62
Compost (compost)	1.2	8.46
Rice husk biochar + compost (rbio + comp)	2.4	4.5∗
Corn cob biochar + compost (cbio + comp)	2.4	4.45∗
Coconut husk biochar (300 °C) + compost (coco300 + comp)	2.4	5.83∗
Coconut husk biochar (700 °C) + compost (coco700 + comp)	2.4	6.04∗
Composted corn cob biochar (cococomp)	1.2	7.75
Composted Rice husk biochar (rcocomp)	1.2	8.99

WSOC = water soluble organic carbon.

∗ WSOC in these treatments were estimated from the WSOC determined from their component biochars and composts, respectively.

In this study, biochar and compost were considered to play different roles in improving soil quality, hence compost and biochar were added at equal amounts in the combined compost and biochar treatments to determine their combined effect on soil quality, soil C stability and N content relative to when they are added singly. Compost was considered as an N-rich amendment that improves soil N and nutrients contents whiles biochar was viewed as a stable C-rich input that enhances soil C stability and soil physical properties.

### 2.3 Laboratory analyses

The moisture content in soil and amendments were determined in an oven at 105 °C for 24 h. The amendments were also analyzed for ash, volatile matter and fixed carbon content by proximate analysis following ASTM standards (D 1762–84) modified by (Mukherjee et al., 2011). Fixed carbon was determined by subtracting the sum of the percentage moisture, volatile matter and the ash contents from 100. Total C and total N were analyzed by dry combustion (Vario EL Elementar Analysesysteme GmbH, Hanau, Germany) after grinding the dried samples. Soil pH was determined with a glass electrode (WTW 192, Ingold) in 0.01 M CaCl_2_ (1:25 w/v). The basal respiration was estimated weekly by titrating 10 ml 0.5 M KOH solution placed inside the beakers with 0.5M HCl. Microbial biomass C (Cmic) was determined by the chloroform fumigation extraction method (Vance et al., 1987). Incubated moist soil (1.2 g) was fumigated at room temperature with ethanol-free CHCl_3_ for 24 h in a desiccator. The fumigated sample and non-fumigated controls were extracted with 24 ml of 0.05 M K_2_SO_4_ by 30 min horizontal shaking and subsequent filtration (Whatman GF/A filters). The supernatant was subject to C and N determination with the Dimatoc 2000 automatic analyzer (Dimatec, Essen, Germany). C_mic_ was calculated as difference between total C extracted from fumigated and non-fumigated treatments, divided by 0.45 (Vance et al., 1987).

The article "Can combined compost and biochar application improve the quality of a highly weathered coastal savanna soil?" was published in 2021. Journal: Heliyon.

Metabolic quotient (qCO2), the ratio of basal respiration and microbial biomass was determined to describe the CO_2_–C produced per unit C_mic_ (Spohn, 2015) while C_mic_/total C ratios were calculated to describe C availability for microbial growth. All results are reported on an oven-dry (105 °C) weight basis. Hot water soluble C contents (WSOC) in the amendments used in the study were determined according to Ghani et al. (2003). A mixture of 1.2 g of each amendment and 24 ml H_2_O were heated for 16 h in a water bath at 80 °C. The mixture was then cooled and shaken for 30 min prior to centrifugation. Then the supernatant was passed through a 0.45 μm filter (Whatman GF/A) and DOC in each mixture was analyzed with a Dimatoc 2000 automatic analyzer (Dimatec, Essen, Germany) to represent their WSOC.

Exchangeable cations and CEC were determined using the ammonium chloride (at pH 7) extraction method. About 2.5 g sample from each treatment was weighed into a 50 ml beaker and 10 ml of the exchange solution was added. The beaker was covered with a watch glass and allowed to stand for 24 h. Percolation was done after 24 h by rinsing the sample with the solution into the filter paper and collecting the filtrate in a 100 ml measuring flask. The percolation lasted about 4 h with approximately 90 ml of the percolate being collected in the flask. The concentrations of the exchangeable cations (Ca^2+,^ Mg^2+^, Na^+^ and K^+^) were measured by Inductively Coupled Plasma Spectroscopy (ICP-OES) and the CEC was calculated as the sum of the exchangeable cations.

### 2.4 Statistical analyses

The statistical analyses were done with the 12th edition of GenStat statistical software. Descriptive analyses, and tests for normality and homogeneity of variances were conducted prior to a one-way analysis of variances (ANOVA). ANOVA was used to test the effects of treatments on soil quality parameters. Pearson's correlation analysis was used to determine whether there were significant interrelationships among the measured properties of the soils. Treatment means were separated by Duncan tests to determine whether or not they were significantly different from each other.

The article "Can combined compost and biochar application improve the quality of a highly weathered coastal savanna soil?" was published in 2021. Journal: Heliyon.

## 3 Results

### 3.1 Basal respiration

The effects of biochar and/or compost application on soil basal respiration are presented in Figure 1a and b.

**Figure 1:** a. Basal respiration rate following the application of sole compost and combined biochar and compost to soil. b. Basal respiration rate following the application of biochar and composted biochar to soil.

The sole compost treatment and all the combined biochar and compost treatments (cbio + comp, rbio + comp, coco300 + comp and coco700 + comp) showed significant (*P* < 0.05) increases in basal respiration above 1 mg CO_2_ m^−2^ h^−1^ (Figure 1a) compared to the sole biochar (cbio, rbio, coco300 and coc700), composted biochar (rcocomp and cococomp) and the control treatments, respectively, which showed basal respiration values below 1 mg CO_2_ m^−2^ h^−1^ (Figure 1b).

In all the treatments, basal respiration was greater on day 7 after incubation than on days 14, 21 and 30, respectively (Figure 1a and b). Among the sole compost and the combined biochar and compost treatments, coco300 + comp, rbio + comp and cbio + comp showed significant increase in basal respiration on day 7, 14 and 21 compared to coco700 and the sole compost. Similarly, in the sole biochar and the composted biochar treatments, rcocomp and cococomp recorded significant increases in basal respiration from day 7 to day 30 compared to rbio, cbio and the control treatments. However, cbio and rbio did not significantly increase basal respiration from day 7 to day 30 after incubation compared to the control.

### 3.2 Effect of biochar and/or compost or composted biochar on selected soil properties

The effects of sole biochar, sole compost, combined compost and biochar or composted biochar additions on soil pH, total organic carbon (TOC), total nitrogen (TN) contents and microbial biomass carbon (MBC) are summarised in Table 3 while their effects on soil total respiration (TR), MBC/TOC, Metabolic quotient (qCO2) and TOC/TR after 30 days of incubation are shown in Table 4, respectively.

**Table 3:** Effects of biochar and/or compost or composted biochar on soil pH, TOC, TN and MBC after 30 days of incubation.

Treatments	pH	TOC (%)	TN (%)	MBC (μg/g)
Control	4.39	0.81 ± 0.03a	0.10 ± 0.00a	62.71 ± 16.53a
Rbio	4.67	1.59 ± 0.56cde	0.14 ± 0.05b	62.96 ± 18.31a
Cbio	4.80	1.55 ± 0.09cde	0.11 ± 0.00ab	68.23 ± 8.33a
coco 300	5.02	1.40 ± 0.02bcd	0.11 ± 0.00ab	72.62 ± 2.27a
coco 700	5.47	1.52 ± 0.02cde	0.10 ± 0.00a	73.98 ± 3.26a
Compost	6.38	1.11 ± 0.05b	0.12 ± 0.00ab	217.63 ± 55.09d
Rcocomp	5.64	1.16 ± 0.03b	0.11 ± 0.00ab	106.50 ± 9.40ab
Cococomp	5.75	1.35 ± 0.04bc	0.11 ± 0.00ab	109.25 ± 6.72ab
rbio + comp	5.98	1.47 ± 0.02cde	0.12 ± 0.00ab	145.64 ± 78.87bc
cbio + comp	6.09	1.76 ± 0.04e	0.12 ± 0.00ab	209.47 ± 16.79d
coco 300 + comp	6.20	1.61 ± 0.02cde	0.13 ± 0.00ab	196.06 ± 23.09cd
coco 700 + comp	6.68	1.70 ± 0.02de	0.12 ± 0.00ab	185.22 ± 33.17cd
***p* value**		<0.001	0.207	<0.001

**LSD (0.05)**		0.279	0.025	53.291

Figures followed by the same letters are not significantly different are P < 0.05.

The article "Can combined compost and biochar application improve the quality of a highly weathered coastal savanna soil?" was published in 2021. Journal: Heliyon.

**Table 4:** Effects of biochar and/or compost or composted biochar on soil total respiration (TR), MBC/TOC, Metabolic quotient (qCO_2_) and TOC/TR after 30 days of incubation.

Treatments	MBC/TOC	TR (mg CO_2_ (m^2^ h^−1^))	MBC/TR (qCO_2_)	TOC/TR
control	77.48 ± 23.34abc	0.65 ± 0.03a	95.93 ± 21.17de	1.25 ± 0.09bc
rbio	39.60 ± 22.86a	0.65 ± 0.02a	96.51 ± 27.59de	2.45 ± 0.92e
cbio	44.07 ± 7.11a	0.64 ± 0.02a	106.20 ± 14.62e	2.40 ± 0.07e
coco300	51.72 ± 2.25ab	0.80 ± 0.07ab	91.12 ± 9.93de	1.76 ± 0.13d
coco700	48.52 ± 1.93ab	0.98 ± 0.04bc	75.29 ± 2.77cd	1.55 ± 0.04cd
compost	195.59 ± 46.88d	3.67 ± 0.14e	59.00 ± 13.49bc	0.30 ± 0.01a
rcocomp	92.17 ± 8.97bc	1.13 ± 0.03cd	94.45 ± 11.08de	1.02 ± 0.04b
cococomp	81.15 ± 7.29abc	1.27 ± 0.07d	86.37 ± 7.22de	1.07 ± 0.08b
rbio + comp	98.83 ± 54.24c	5.14 ± 0.06g	28.32 ± 15.32a	0.29 ± 0.00a
cbio + comp	118.75 ± 11.66c	5.46 ± 0.12h	38.30 ± 2.29ab	0.32 ± 0.01a
coco 300 + comp	121.70 ± 13.22c	5.57 ± 0.35h	35.39 ± 6.11ab	0.29 ± 0.02a
coco 700 + comp	108.85 ± 20.52c	4.43 ± 0.30f	41.72 ± 5.96ab	0.39 ± 0.03a
***p* value**	<0.001	<0.001	<0.001	<0.001

**LSD (0.05)**	41.080	0.246	22.815	0.456

Figures followed by the same letters are not significantly different are P < 0.05.

#### 3.2.1 Soil pH, total organic carbon (TOC) and total nitrogen (TN)

Application of biochar and/or compost or composted biochar increased soil pH by 0.28–2.29 pH units (Table 3). Sole compost and composted biochar addition increased soil pH more than sole biochar application. The combined rice husk or corn cob biochar and compost amended soils showed higher soil pH values than their corresponding sole biochar and composted biochar treatments.

TOC in all the amended soils was greater than the control (Table 3). TOC in the sole biochar and combined biochar and compost treatments was greater than their corresponding sole compost and composted biochar treatments except for cococomp. In this study, sole compost application increased TOC by 37% compared to the control; combined application of biochar and compost increased TOC by 81.5–117.3% compared to the control; while additions of composted rice husk and corn cob biochars increased TOC by 43.2 and 66.7 %, respectively. However, regardless of the feedstock, addition of biochar together with compost did not increase TOC more than the sole application of biochar. TN found in all the treatments were not statistically different from the control except for rbio which increased TN by 40%.

The article "Can combined compost and biochar application improve the quality of a highly weathered coastal savanna soil?" was published in 2021. Journal: Heliyon.

#### 3.2.2 Microbial biomass carbon (MBC) and ratio of MBC to TOC (MBC/TOC)

MBC in all the sole biochar and composted biochar treatments were similar to the control. However, when biochar and compost were applied together, MBC was increased by 82.9–146.8 μg g^−1^ compared to the control. Also, sole application of compost increased MBC more than the corresponding composted biochars. The ratio of MBC to TOC in all the treatments were similar to the control except for the sole compost treatment. Applying compost alone increased MBC/TOC by 152.4%. Although applying biochar together with compost increased MBC/TOC more than their corresponding sole biochar treatments, differences between them and the control were not statistically significant.

#### 3.2.3 Total respiration (TR) and metabolic quotient (qCO_2_) (MBC/basal respiration)

Total respiration was calculated by summing up the basal respiration measured on days 7, 14, 21 and 30 for each treatment. The sole biochar treatments showed no significant differences in TR compared to the control treatment except for coco 700 (Table 2). TR in the amended soils followed the decreasing order: combined biochar and compost > sole compost > composted biochar > sole biochar > control. Among the combined biochar and compost treatments, coco300 + comp gave the highest TR value of 5.57 mg CO_2_ m^−2^ hr^−1^, which was also the highest among all the treatments. Microbial quotient (qCO_2_) was lower in the sole compost and the combined biochar and compost treatments compared to the control. However, qCO_2_ for the sole biochar and the composted biochar treatments were not statistically different from the control.

#### 3.2.4 Cation exchange capacity (CEC)

CEC in all the treatments were significantly higher relative to the control (Figure 2). The application of biochar together with compost increased CEC more than biochar applied alone. CEC in the composted biochar treatments were similar to those in the sole compost treatments but these were higher than those found in their corresponding combined compost and biochar treatments.

**Figure 2:** Effect of biochar and/or compost application on CEC.

#### 3.2.5 Available nitrogen (${\text{NH}}_{4}^{+}$ –N and ${\text{NO}}_{3}^{-}$ –N)

The effect of biochar and/or compost application on available N (${\text{NH}}_{4}^{+}$ –N and ${\text{NO}}_{3}^{-}$ –N) contents are presented in Figures 3 and 4, respectively. Inorganic ${\text{NH}}_{4}^{+}$ –N concentrations in all the amendments were lower (*P* < 0.05) than the control except for rbio and cbio (Figure 3). The ${\text{NH}}_{4}^{+}$ –N concentrations in the sole biochar amended soil were higher than their corresponding combined biochar and compost treatments. However, no significant differences were observed among the sole compost, composted biochar and the combined compost and biochar treatments.

The article "Can combined compost and biochar application improve the quality of a highly weathered coastal savanna soil?" was published in 2021. Journal: Heliyon.

**Figure 3:** Effect of biochar and/or compost application on NH_4_–N contents.

**Figure 4:** Effect of biochar and/or compost application on NO_3_–N.

Inorganic ${\text{NO}}_{3}^{-}$ –N concentrations were higher in the sole compost, composted biochar and the sole biochar treatments as compared to the control (Figure 4). The ${\text{NO}}_{3}^{-}$ –N concentrations in the sole biochar amended soil were higher than their corresponding combined biochar and compost treatments. The highest ${\text{NO}}_{3}^{-}$ –N concentrations was recorded in the sole compost treatment followed by the composted biochar treatments.

#### 3.2.6 Biochar and compost mineralisation (% SOC and CO_2_ release)

C mineralized in biochar and/or compost amended soils are presented in Figure 5, and CO_2_ release following biochar and/or compost application are shown in Figure 6.

**Figure 5:** Effect of biochar and/or compost application on C mineralization.

**Figure 6:** Effect of biochar and/or compost application on CO_2_ release.

C mineralized from the sole compost treatment was significantly greater than all the other treatments (Figure 5), but no significant differences occurred in the C mineralized from the sole biochar and composted biochar amended soils, which were similar to the control. Combined application of biochar and compost caused greater CO_2_ release than sole compost application (Figure 6). CO_2_ release from the sole compost was greater than CO_2_ release from the sole biochar treatments. Across the treatments, CO_2_ release from all the sole biochar treatments were similar to the control except for coco 700.

#### 3.2.7 Correlation matrix showing relationships between the soil properties

A matrix showing the co-efficient of correlation relationships between selected soil quality indicators considered in this study are shown in Table 5. The correlation co-efficient indicate that pH positively correlated with CEC, TR and MBC but negatively correlated with ${\text{NH}}_{4}^{+}$ –N and qCO_2_. TOC and TN correlated positively with TR and negatively with ${\text{NH}}_{4}^{+}$ –N and qCO_2._ TR and MBC correlated positively with each other but both correlated negatively with ${\text{NH}}_{4}^{+}$ –N, NO_3_–N and qCO_2._

**Table 5:** Pearson correlation matrix.

Parameter	NO_3_–N	NH_4_–N	CEC	qCO_2_	TR	MBC	C/N	TOC	TN
pH	0.056 ns	-0.778∗∗	0.608∗∗	-0.746∗∗	0.802∗∗	0.823∗∗	0.237 ns	0.324 ns	0.218 ns
TN	-0.272 ns	0.012 ns	0.324 ns	-0.440∗∗	0.341∗	0.232 ns	0.011 ns	0.634∗∗	
TOC	-0.465∗∗	-0.115 ns	0.288 ns	-0.471∗∗	0.391∗	0.202 ns	0.778∗∗		
C/N	-0.333∗	-0.162 ns	0.141 ns	-0.234 ns	0.199 ns	0.055 ns			
MBC	-0.057 ns	-0.552∗∗	0.455∗∗	-0.610∗∗	0.831∗∗				
TR	-0.378∗	-0.528∗∗	0.285 ns	-0.896∗∗					
qCO_2_	0.343∗	0.547∗∗	-0.263 ns						
CEC	0.447∗∗	-0.499∗∗							
NH_4_–N	-0.335∗								

ns: not significant.

∗∗Correlation is significant at the 0.01 level.

∗Correlation is significant at the 0.05 level.

The article "Can combined compost and biochar application improve the quality of a highly weathered coastal savanna soil?" was published in 2021. Journal: Heliyon.

## 4 Discussion

In this study, sole biochar additions did not significantly increase basal respiration compared with the control (Figure 1b). This finding is in good agreement with Zavalloni et al. (2011) who found that respiration rates in soil treated with coppiced woodland-derived biochar were not significantly different from the control soil. Previous authors (Méndez et al., 2013; Thies et al., 2009) opined that low CO_2_ emissions from biochar amended soils can be attributed to chemisorptions of the respired CO_2_ on the biochar surface. Basal respiration from the combined biochar and compost, sole compost and composted biochar treatments, respectively, were greater than the sole biochar treatments (Figures 1a and 1b). The higher basal respiration found in the sole compost, combined biochar and compost and the composted biochar treatments is an indication of increased biological activity in those treatments. Additionally, the study showed rather unexpectedly that mixing compost with very inert biochars (rbio and cbio) greatly increased mineralization, with the lowest effects occurring rather with the most labile biochar (coco700). The underlying reason for this observation is not clear but it raises the critical questions whether the biochar removed some toxic compounds or provided additional nutrients, which would have stimulated the mineralization process. Further studies need to be done to establish the mechanisms underpinning this observation.

The differences in basal respiration observed in the compost and/or biochar amended soils can be attributed to their varying labile carbon contents as suggested by Méndez at al. (2013). Benito et al. (2005) reported that, the high water soluble carbon content of compost can stimulate microbial activity, resulting in increased carbon dioxide (CO_2_) fluxes and soil organic matter (SOM) decomposition through priming effect. The coconut husk biochars (coco300 and coco700) had higher water-soluble carbon contents than the corn cob and rice husk biochars (cbio and rbio), respectively (Table 2). Although the coconut husk biochar pyrolysed at 700 °C (coco 700) showed higher WSOC than coconut husk biochar pyrolysed at 300 °C (coco 300), it did not result in a higher MBC (Table 3).

The article "Can combined compost and biochar application improve the quality of a highly weathered coastal savanna soil?" was published in 2021. Journal: Heliyon.

The results also revealed that co-composting greatly reduced the labile C contents of the product, which also reflected in the MBC. Sole biochar amended soils showed lower MBC than the sole compost and the combined compost and biochar treatments, respectively, but, MBC in the sole biochar and composted biochar treatments were similar (Table 3). The result is in agreement with Liu et al. (2004) who observed no effect of corn cob biochar on MBC in a laboratory experiment in which corn cob pyrolysed at 550 °C had been incorporated in a sandy loam at 15 t ha^−1^ Méndez et al. (2013) and Thies et al. (2009) argued that the electrical conductivity, metal and phenolic substances of biochar can slow down soil microbial activity reducing the respired CO_2_. In contrast, Khan et al. (2014) reported that many studies have shown increased MBC with biochar additions. According to Kuzyakov et al. (2009), a small fraction of labile C mineralized within a short period after biochar application can stimulate microbial activity in soils (Quilliam et al., 2013), which is indicative that biochar supply soil microbes with labile C (Gomez et al., 2014) to enhance their activity and efficiency to induce soil C mineralization or degradation (Luo et al., 2011). In this study, sole applications of corn cob, rice husk or coconut husk biochars did not significantly increase MBC in the soil. Jindo et al. (2012) reported that low MBC in biochar amended soils was due to their low labile C contents.

According to Chen et al. (2005), soil microorganisms greatly depend on soil organic matter as their sources of labile C and so a decrease in SOC is likely to result in low soil microbial biomass. Thus, the relatively higher MBC found in the sole compost and the combined compost and biochar amended soils are attributable to their greater organic C contents (Wang and Yang, 2007). Farrell et al. (2009) reported that MBC is a useful indicator of soil C stabilization while Bierdeman and Harpole (2013) posited that increased MBC is an indication of higher availability of labile C inputs. In this study, the trend found in MBC contents in the amended soils was similar to that observed for the basal respiration. Thus, the low MBC and basal respiration observed in the sole biochar amended soils are reflections of low microbial activity. Additionally, the higher, MBC found in the combined compost and rice husk or corn cob biochar treatments compared with their corresponding composted biochars, suggest that decomposable C may have been stabilized in the composted biochars.

The article "Can combined compost and biochar application improve the quality of a highly weathered coastal savanna soil?" was published in 2021. Journal: Heliyon.

MBC/SOC ratio shows substrate availability and the portion of total soil carbon immobilized in microbial cells (Yang et al., 2010). Therefore, the relatively lower MBC/SOC ratios in the sole biochar amended soils (Table 4) may be attributed to the inhibition of microbial C immobilization, while a relatively higher MBC/SOC ratio in the sole compost amended soil indicates a stimulation of microbial C immobilization. The potentially higher amount and diversified C contents in the combined compost and biochar and composted biochar treatments could have resulted in higher labile carbon availability.

Soil MBC/SOC ratio, or microbial quotient, has been widely used as an indicator of future changes in organic matter due to modifications of soil conditions (Sparling et al., 1992). Furthermore, Joergensen (1999) reported that this ratio has been used as an index to compare soil quality across soils with varying organic matter contents. Thus, the MBC/SOC ratio mirrors the relationship and interactions between the MBC and SOC (Yang et al., 2010). The large amounts of recalcitrant carbon in biochar amended soils can slow down the rate of decomposition and transformation of particulate organic matter into mineral soil component (Leckie et al., 2004). This is evidenced in this study by the relatively lower TON and basal respiration found in the sole biochar amended soils.

Previous studies reported positive correlations between litter layer C/N ratio and respiration (Spohn, 2015; Michel and Matzner, 2003). In this study, a positive correlation was found between soil C/N ratio and basal respiration at day 7 but this was not statistically significant. Spohn and Chodak (2015) found a positive correlation between qCO_2_ and soil C/N ratios in beech, spruce, and mixed forests. Three reasons have been proffered for the observed relationships between C/N ratio and qCO_2_ and basal respiration. First, Craine et al. (2007) argued that microorganisms break down readily available C in order to gain the energy needed to acquire N from more recalcitrant forms of organic matter or access the N incorporated in organic compounds. However, microorganisms in N-limited soils have very limited capacity to invest N into the production of exoenzymes and release them to acquire C.

Secondly, Birt and Bonnett (2018), and Manzoni et al. (2010) attributed the relationship to overflow respiration, which implies that microorganisms uncouple respiration from energy production and only respire C to dispose it off. However, the relevance of microbial overflow respiration in ecosystems has been questioned (Hessen and Anderson, 2008) on the basis that N is needed to maintain the proteins of the respiratory chain so as to dispose off C via respiration (Hessen and Anderson, 2008). Finally, Carreiro et al. (2000), Michel and Matzner (2003) and Gallo et al. (2004) explained that the oxidative enzymes activities involved in the degradation of aromatic compounds, decreases with increasing N concentration. Thus, decreased lignolytic activity may decrease microbial respiration in litter with low C/N ratios (Carreiro et al., 2000; Eiland et al., 2001).

The article "Can combined compost and biochar application improve the quality of a highly weathered coastal savanna soil?" was published in 2021. Journal: Heliyon.

Higher qCO_2_ in a treatment suggests that more C is probably channelled into the energy metabolism and a lower efficiency in microbial biomass C formation. Some authors have argued that low qCO_2_ rates in less stressed ecosystems indicates high microbial activity and efficiency, leading to a higher organic matter decomposition and C mineralization. MBC values found in this study indicate that the efficiency of microbial C formation was relatively lower in the sole compost treatment than in the combined biochar and compost treatments. Furthermore, lower water-soluble C was found in the sole biochar amended soils than the sole compost treatment. Therefore, the higher MBC and basal respiration observed in the sole compost treatment compared to the sole biochar treatments was not unexpected. However, it appears that basal respiration was disproportionately greater than MBC in the sole compost amended soils, resulting in their relatively lower qCO_2_ values.

This study showed that biochar and/or compost additions increased soil pH above that of the control soil. Méndez et al. (2012) observed a pH increment in a Haplic cambisol after the addition of sewage sludge-derived biochar. Kloss et al. (2014) also found slight increment of soil pH (0.3 units) in an acid soil after application of woodchip-derived biochar, whereas Jien and Wang (2013) observed a significant increase (from 3.9 to 5.1) in an Ultisol following addition of wild lead tree, and waste wood biochar. It must be pointed out that pH of 6.6–7.3 is favourable for microbial activities that contribute to the availability of nitrogen, sulphur, and phosphorus in soils (USDA FS, 1998), and a pH value exceeding 10 can have negative effects on soil nutrient availability.

Results from this study indicated that TOC in all the amended soils were greater than the control. This is in agreement with previous studies (Angst et al., 2014; Kimetu and Lehmann, 2010; Xie et al., 2013), which reported increased total SOC following the applications of various biochar types. The significantly higher TOC observed in the combined biochar and compost treatments, reflected the high C concentration in the amendment C originally added to the soil during incubation.

The article "Can combined compost and biochar application improve the quality of a highly weathered coastal savanna soil?" was published in 2021. Journal: Heliyon.

In this study, it was observed that sole biochar and sole compost application increased TON by 12–27%, but TON in the combined biochar and compost treatments were greater than their corresponding composted biochar treatments. This result is in accordance with Xie et al. (2013) who reported that biochar addition increased soil N contents. In contrast, Lehmann and Joseph (2009) reported that pure biochar does not directly enrich the soil with nutrients. Lehmann et al. (2003) argued that biochar addition may elevate soil C/N ratio, thereby reducing N mineralization. Following the ideas of Schulz and Glaser (2012), we hypothesize that composting biochar can have a stabilizing effect on early decomposable components of the compost. This will lead to a relatively lower N contents in the composted biochar treatments than the combined compost and biochar treatments.

Berglund et al. (2004) and De Luca et al. (2002) explained that notwithstanding the low N content of many biochars, their application may result in net nitrification due to the labile C they release and their ability to increase soil pH. This observation is confirmed by, the greater TON observed in the combined biochar and compost treatments. However, the results in this study did not clearly provide any evidence of a positive priming effect. Yao et al. (2011) reported that biochar application can negatively affect nitrification, particularly, if the pH increases to values of 10 or above. In this study, none of the amendments increased soil pH to values above 10 and so no net effect on nitrification could have occurred. Biochar application increased soil CEC but, CEC in sole biochar treatments were lower than in the sole compost, combined biochar and compost and the composted biochar treatments, which is indicative of the low inherent CEC of biochar compared to compost (Lehmann, 2007).

## 5 Conclusions

In agreement with our hypothesis, the study has demonstrated that combined application of N-rich compost and C- rich biochar, and composted biochar enhanced soil quality through increased TOC, TON, MBC, CEC and soil pH compared to the control. The study also showed that sole application of biochar can lower basal respiration, thereby stabilizing soil C compared to sole compost application. Furthermore, the study showed that regardless of whether compost was added solely or in combination with biochar, its addition to highly weathered soils increased the efficiency at which C was converted into MBC.

## Declarations

### Author contribution statement

Kwame Agyei Frimpong: Conceived and designed the experiments; Performed the experiments; Analyzed and interpreted the data; Wrote the paper.

The article "Can combined compost and biochar application improve the quality of a highly weathered coastal savanna soil?" was published in 2021. Journal: Heliyon.

Emmanuel Abban-Baidoo: Performed the experiments; Analyzed and interpreted the data; Wrote the paper.

Bernd Marschner: Conceived and designed the experiments; Contributed reagents, materials, analysis tools or data.

### Funding statement

This work was supported by TWAS-DFG and the Ruhr University of Bochum.

### Data availability statement

Data included in article/supplementary material/referenced in article.

### Declaration of interests statement

The authors declare no conflict of interest.

### Additional information

No additional information is available for this paper.
